# Comparison of Diagnostic Efficacy among Transvaginal Sonography, Transabdominal Sonography, and 3.0 T Magnetic Resonance Imaging in Early Cesarean Scar Pregnancy

**DOI:** 10.1155/2022/9714369

**Published:** 2022-01-25

**Authors:** Ke Wang, Fangbin Jing

**Affiliations:** ^1^Department of Ultrasound, Zibo First Hospital, Zibo 255200, Shandong Province, China; ^2^Department of Ultrasound Medicine, Laiyang Central Hospital of Yantai City, Yantai 265200, Shandong Province, China

## Abstract

**Objective:**

To compare the diagnostic efficacy among transvaginal sonography (TVS), transabdominal sonography (TAS), and 3.0 T magnetic resonance imaging (MRI) in early cesarean scar pregnancy (CSP).

**Methods:**

The clinical data of 65 patients initially diagnosed with CSP in our hospital from November 2019 to November 2020 were selected for the retrospective analysis, and all patients received TVS, TAS, and 3.0 T MRI. Taking the pathological findings as the “gold standard”, the diagnostic efficacy of different diagnostic modalities in early CSP was compared.

**Results:**

In terms of the AUC value, the result was 3.0 T MRI > TVS > TAS, and among the three diagnosis methods, 3.0 T MRI had the highest diagnostic specificity, and TVS and 3.0 T MRI had the highest sensitivity; other than intragestational hemorrhage, the detection rates of other signs of disease by TVS and TAS were significantly higher than 3.0 T MRI (*P* < 0.05).

**Conclusion:**

3.0 T MRI has better diagnostic efficacy in early CSP than TVS and TAS, while TVS and TAS work better in diagnosing uterine bleeding, plumule, yolk sac, and fetal heartbeat than 3.0 T MRI. The results are more beneficial to the guidance on selecting treatment modalities.

## 1. Introduction

Cesarean scar pregnancy (CSP) is a type of heterotopic pregnancy at a special site in pregnant women who have undergone cesarean section (C-section) before, which is mainly manifested by embryos implanted at the lower uterine segment where the incision scar is located and is one of the long-term complications of C-section [1, 2]. The specific etiology remains unclear, and it is speculated that it may be related to the history of C-section or other surgery on the endometrium, which changes the environment of the local uterine cavity and results in the difficulty of the zygote to implant on the anterior and posterior walls of the uterine body, so the zygote migrates to the scar site for growth and development, and thereby leading to CSP. Recently, the incidence of CSP has increased year by year due to the increased rate of C-sections. Because the CSP has no specific manifestation, it is prone to clinical erroneous diagnosis and missed diagnosis, and failure to timely diagnose and take appropriate care measures will lead to major bleeding, uterine perforation, rupture, and other serious complications in patients [3–5]. At present, inquiring the medical history, imaging, and pathological examination are the common methods in clinic to confirm the diagnosis, and surgical exploration is a commonly used examination method in CSP, which is clinically regarded as the examination “gold standard”, but it is risky and difficult to promote the application in primary hospitals. Therefore, imaging examination has an increasing role in diagnosing early CSP [6]. Ultrasonography is valuable for the diagnosis of CSP, which clearly shows the blood supply to the pregnant decidua from the uterine scar and indicates the embryo implantation site, but it is difficult for the diagnosis of atypical CSP because of its high operator requirement and inability to show the morphology of the gestational sac and its relationship with surrounding tissues, which may lead to missed diagnosis and erroneous diagnosis [7, 8]. Magnetic resonance imaging (MRI) technique has good contrast in soft tissue examination and is capable of multidirectional imaging, and its diagnostic efficacy has been demonstrated in early benign and malignant lesions of the breast, ovarian cancer, fibromas of the follicular membrane, and other diseases [9, 10]. 3.0 T MRI shows dynamic changes of human tissue structures more clearly because of its high imaging speed, high signal-to-noise ratio, and high image resolution, but such diagnostic modality has a relatively long scanning time and many artifacts. This study is expected to provide a more clinical basis for diagnosis and treatment of CSP by comparing the characteristics of transvaginal sonography (TVS), transabdominal sonography (TAS), and 3.0 T MRI in diagnosing early CSP and analyzing their advantages and disadvantages.

## 2. Materials and Methods

### 2.1. General Data

The clinical data of 65 patients initially diagnosed with CSP in our hospital from November 2019 to November 2020 were selected for the retrospective analysis, and the study met the World Medical Association Declaration of Helsinki (2013) [11]. Inclusion criteria: ① patients had undergone more than one C-section before and were 22 to 45 years old, and their clinical symptoms included amenorrhea, an irregular small amount of vaginal bleeding, and mild abdominal pain; ② 3–8 weeks after cessation of menstruation, elevated human chorionic gonadotropin (*β*-HCG) value was found via blood examination; and ③ patients had completed clinical imaging data. Exclusion criteria: ① puerpera had other types of heterotopic pregnancy (tubal pregnancy, abdominal pregnancy, cervical pregnancy, etc.); ② patients were complicated with other gynecological diseases that affected the diagnosis of CSP; ③ patients had an allergic constitution and could not accept MRI; and ④ patients were complicated with reproductive system malignancies or had mental diseases.

### 2.2. Methods

The examination instrument selected was the DU8-M2 color Doppler ultrasonic tester (manufactured: Xuzhou Ruihua Electronic Science & Technology Development Co., Ltd.), and the probe frequency for TVS and TAS was 5–9 MHz and 1–5 MHz, respectively. First, the TAS was performed. Patients filled their bladder before examination and then lied in spine position, coupling agent was applied to their lower abdomen, and the probe was placed on their abdomen for exploration to carefully observe whether the size and shape of the uterus, the presence or absence of abnormal adnexal mass, gestation sac in the uterine cavity, abdominal or pelvic hydrops, and echogenicity inside internal uterine cavity were associate with the uterine scar. After that, patients emptied their urine and received TVS examination in lithotomy position, an ultrasonic probe wrapped with a sterile condom was put into their cavity via vagina for full-range scanning, routine examination of the uterus, pelvic cavity, and bilateral appendixes, and observation of size, location, and echogenicity of gestation sac, to find out whether they were related to C-section scar [6, 12]. Meanwhile, attention should be paid to observe whether there was a bulging mass or the presence or absence of a gestational sac at the incision of the uterine site, the specific location and morphology of the mass and gestational sac, and the trophoblast flow signal, and to measure the size of the gestational sac as well as the thickness of the muscular layer of the anterior uterine wall.

3.0 T MRI: patients were in spine position and asked to control their breathing; the MAGNETOM Skyra 3.0 T MRI superconducting scanner (manufactured: Siemens AG) and body phased-array coil was used to perform routine scanning with the following scanning sequences. Turbo spin echo (TSE): T1WI (TR 522 ms, TE 21 ms), T2WI (TR 3,700 ms, TE 93 ms), slice thickness 5 mm, slice gap 1.0 mm, matrix 320 × 320, the field of view (FOV) 350 mm × 350 mm; fat-saturated T2WI sagittal sequence: TR 5,000 ms, TE 93 ms, slice thickness 5 mm, slice gap 1.0 mm, matrix 320 × 320, and FOV 260 mm × 260 mm. The images were analyzed and observed by 2 experienced radiologists.

### 2.3. Observation Index

Taking the results of pathological diagnosis as the “gold standard,” the diagnostic efficacy of TAS, TVS, and 3.0 T MRI examinations was compared.

### 2.4. Statistical Methods

The data obtained in this study were analyzed by SPSS 26.0, the relevant accuracy rates of diagnosing CSP via 3 imaging modalities were examined by X^2^ test, and differences were considered statistically significant at *P* < 0.05.

## 3. Results

### 3.1. Comparison of Results of Different Imaging Examinations and Pathological Diagnosis

The results of pathological diagnosis showed that 54 cases were positive and 11 cases were negative for CSP. For comparison of results of the three imaging diagnosis modalities and pathological diagnosis; see Tables 1–3.

### 3.2. Comparison of Diagnostic Efficacy among Different Imaging Diagnosis Modalities

The AUC values of diagnosing CSP via TAS, TVS, and 3.0 T MRI were 0.727, 0.776, and 0.844, respectively, and among them, 3.0 T MRI had the highest diagnostic specificity, and TVS and 3.0 T MRI had the highest sensitivity (Table 4).

### 3.3. Comparison of Different Diagnosis Modalities in Detecting Signs of Disease

Other than intragestational hemorrhage, the detection rates of other signs of disease by TVS and TAS were significantly higher than 3.0 T MRI (*P* < 0.05) Table 5.

### 3.4. Analysis of ROC Curves of Different Imaging Diagnosis Modalities

For analysis of ROC curves of the three imaging diagnosis modalities, see Figure 1.

## 4. Discussion

CSP is a special ectopic pregnancy manifested by the implantation of the gestational sac at the incision of a C-section. At the early stage of CSP, there are no specific clinical manifestations, which largely increase the difficulty of diagnosis, and with the progress of pregnancy, the CSP will easily trigger uterine rupture, major bleeding, and other symptoms, seriously threatening the life safety of patients [13]. Ultrasound diagnosis is a common diagnostic modality for CSP, which launches an ultrasound beam to the human body to produce reflections at different demarcations of acoustic resistance in various tissues, and then the reflected echoes are accepted by the probe and then reconstituted into a sonogram for diagnosis. It is easy to perform, inexpensive and noninvasive, and the application of color Doppler ultrasound has obviously improved the reference value of ultrasound diagnosis [14]. The ultrasound diagnosis enables precise measurement of the physiological tissue structure and morphology in patients, with the diagnostic value that has been proven in diseases including adenomyosis and primary fallopian tube cancer [15]. The thickness of the muscle layer in the lower segment of the anterior uterine wall is currently a common index for the clinical diagnosis of CSP, which can fully reflect the damage situation at the uterine scar [16]. The TVA and TAS are two common modalities of ultrasound diagnosis to provide effective and important information for the treatment and prognosis of patients. With the development of ultrasound diagnosis technology, the TVA and TAS can detect early ectopic pregnancy and now have become the effective means to assist clinical diagnosis [5, 17, 18]. However, ultrasound diagnosis is susceptible to factors such as intestinal gas in patients and physicians' skill levels. MRI, a biological magnetic spin imaging technique, uses the characteristics of spin motion of the nucleus and generates a signal within the external magnetic field after being excited by radiofrequency pulses, then the signal is detected and entered into a computer for processing and transforming into images on-screen. As a multiplanar and multisequence imaging, the MRI has the characteristics such as high spatial resolution, high soft-tissue resolution, and high blood flow sensitivity, and can clearly show the location of the gestational sac in the lower uterine segment and accurately measure the thickness of the gestational sac and the anterior muscular layer, which has unique advantages in assessing the relationship with pelvic visceral structures and the depth of implanted scars [19].

The study results showed that compared with 3.0 T MRI, the AUC value was lower in TVS and TAS in diagnosing the CSP, demonstrating that 3.0 T MRI had higher diagnostic efficacy in confirming early CSP. Further analysis found that the AUC value of TVS was higher than that of TAS, and the reasons might be as follows: although the TAS was able to display the relationship between CSP position and the lower uterine segment as a whole and was convenient to observe the uterine corpus and cervix comprehensively, it confirmed the diagnosis using the principle of large interface reflection [20], hence it was vulnerable to factors such as bladder filling degree, abdominal wall thickness and intestinal gas, which led to sonography showing insignificant near-field echo, making it difficult to accurately measure the thickness between the bladder and the gestational sac, and thus resulting in missed diagnosis and erroneous diagnosis. In addition, compared with TAS, the TVS examination had significantly higher ultrasound probe frequency and higher resolution of the images, which, combined with the fact that the TVS could get more close to pelvic floor organs, would not be disturbed by some factors such as bowel gas and obesity, so the environment inside the uterus, the morphology, and location of the gestational sac, the blood flow signal, etc. could be observed clearly for making a more precise judgment [21]. Imaging and diagnosis with 3.0 T MRI is a new imaging modality in recent years, which is widely used with the continuous advancement of technology and the continuous updating of equipment. Compared with ultrasound diagnosis, 3.0 T MRI enables full range, multiangle as well as multisequence imaging with higher resolution for soft tissue, accurate visualization of the location of the gestational sac, clearer visualization of the relationship between the lesion and the scar of C-section, presenting more obvious advantages in inspection and display for the tissues of pelvic organs [22]. On the other hand, 3.0 T MRI can also find the bleeding phenomenon in the uterine cavity at the local rupture of the myometrium, which is unparalleled by ultrasound diagnosis [23], thereby confirming that 3.0 T MRI has a high clinical application value in the diagnosis of early CSP. In addition, the diagnostic advantage of ultrasound was more prominent in the comparison with the pathological findings, which was due to the fact that 3.0 T MRI is more sensitive to the movement of body parts and prone to artifacts in diagnosis.

## 5. Conclusion

In conclusion, 3.0 T MRI has high diagnostic efficacy in early CSP diagnosis, and its effect is better than that of TVA and TAS, which is beneficial for physicians to carry out observation and develop treatment regimens, demonstrating its role in improving the prognostic effect. Shortcomings of this study: the included sample size was limited, and the findings still need more multicentered studies with large samples for further confirmation; in addition, the quantitative comparative analysis between the lesion and normal myometrium was not performed in this study, so it needs to be more deeply and meticulously explored in the future work.

## Figures and Tables

**Figure 1:** Analysis of ROC curves of different imaging diagnosis modalities. (a, b, c) the ROC curve of TAS, TVS, and 3.0 T MRI, respectively, diagnosing CSP; and the horizontal axes and vertical axes were the specificity (%) and sensitivity (%), respectively.

**Table 1:** Comparison of results of TAS and pathological diagnosis (*n*).

TAS	Results of pathological diagnosis		Total
	Positive	Negative	
Positive	47	3	50
Negative	7	8	15
Total	54	11	65

**Table 2:** Comparison of results of TVS and pathological diagnosis (*n*).

TVS	Results of pathological diagnosis		Total
	Positive	Negative	
Positive	49	2	51
Negative	5	9	14
Total	54	11	65

**Table 3:** Comparison of results of 3.0 T MRI and pathological diagnosis (*n*).

3.0 T MRI	Results of pathological diagnosis		Total
	Positive	Negative	
Positive	50	2	52
Negative	4	9	13
Total	54	11	65

**Table 4:** Comparison of diagnostic efficacy among different imaging diagnosis modalities.

Diagnosis modality	AUC value	Specificity	Sensitivity	95%CI	SE
TAS	0.727	61.11	94.74	0.638–0.817	0.046
TVS	0.776	68.75	96.43	0.693–0.861	0.043
3.0 T MRI	0.844	73.33	96.43	0.768–0.920	0.039

**Table 5:** Comparison of results of different diagnosis modalities and pathological diagnosis [*n* (%)].

Diagnosis modality	Uterine bleeding	Plumule	Yolk sac	Fetal heartbeat	Intragestational hemorrhage
TAS	33 (84.62)^*∗*^	21 (84.00)^*∗*^	25 (83.33)^*∗*^	12 (70.59)^*∗*^	24 (66.67)^*∗*^
TVS	35 (89.74)^*∗∗*^	20 (80.00)^*∗∗*^	24 (80.00)^*∗∗*^	13 (76.47)^*∗∗*^	22 (61.11)^*∗∗*^
3.0 T MRI	6 (15.38)	5 (20.00)	7 (23.33)	2 (11.76)	32 (88.89)
Pathological diagnosis	39	25	30	17	36

*Note.* ^*∗*^Significant difference between TAS and 3.0 T MRI (*P* < 0.05); ^*∗∗*^significant difference between TVS and 3.0 T MRI (*P* < 0.05).

## Data Availability

The data used to support the findings of this study are available on reasonable request from the corresponding author.
